The article "An Optimized Method for Skin Cancer Diagnosis Using Modified Thermal Exchange Optimization Algorithm" was published in 2021. Journal: Comput Math Methods Med.

# An Optimized Method for Skin Cancer Diagnosis Using Modified Thermal Exchange Optimization Algorithm

**DOI:** 10.1155/2021/5527698

**Published:** 2021-06-18

**Authors:** Liu Wei, Su Xiao Pan, Y. A. Nanehkaran, V. Rajinikanth

**Affiliations:** ^1^Gannan University of Science & Technology, Ganzhou, Jiangxi 341000, China; ^2^Ganzhou 851, Ganzhou, Jiangxi 341000, China; ^3^School of Informatics, Xiamen University, Xiamen, 361005 Fujian, China; ^4^Department of Electronics and Instrumentation Engineering, St. Joseph's College of Engineering, Chennai 600119, India

## Abstract

Skin cancer is the most common cancer of the body. It is estimated that more than one million people worldwide develop skin cancer each year. Early detection of this cancer has a high effect on the disease treatment. In this paper, a new optimal and automatic pipeline approach has been proposed for the diagnosis of this disease from dermoscopy images. The proposed method includes a noise reduction process before processing for eliminating the noises. Then, the Otsu method as one of the widely used thresholding method is used to characterize the region of interest. Afterward, 20 different features are extracted from the image. To reduce the method complexity, a new modified version of the Thermal Exchange Optimization Algorithm is performed to the features. This improves the method precision and consistency. To validate the proposed method's efficiency, it is implemented to the American Cancer Society database, its results are compared with some state-of-the-art methods, and the final results showed the superiority of the proposed method against the others.

## 1. Introduction

Cancer, as a difficult disease to treat, has long occupied the human mind [1]. Cancer occurs when cells in a part of the body grow uncontrollably, divide rapidly, invade different tissues in the body, and spread throughout the body [2]. A set of these uncontrollable cells is called a tumor [3]. One of the deadliest sorts of cancers is skin cancer. Skin cancer has grown significantly over the past decades, and the importance of its early treatment is increasing day by day [4].

Melanoma is the third most common type of skin cancer and one of the malignant cancers. Melanoma is also referred to as malignant melanoma, which changes the color of the skin due to the abnormal function of pigment-producing cells. The disease is formed by the accumulation of melanin granules and its spread to the outermost layer of the skin. Despite significant mortality, melanoma is often treatable in the early stages of diagnosis. At the same time, distinguishing between melanoma and other benign moles in the early stages of development is a challenging task, even for dermatologists. Melanoma is known as the 19^th^ prevalent cancer in men and women. There were about 300,000 new cases in 2018.

The article "An Optimized Method for Skin Cancer Diagnosis Using Modified Thermal Exchange Optimization Algorithm" was published in 2021. Journal: Comput Math Methods Med.

The data gathered by the World Health Organization (WHO) in 2018 showed that there were 17852 melanoma cases in the United Kingdom [5]. This organization predicted that the number of melanoma cases will grow by 9% to 19513 with deaths growing by 13% to 3119 by 2025.The growth of skin cancer begins when damage to skin cells (often caused by ultraviolet light) causes mutations that rapidly multiply in skin cells and form malignant tumors.

Normally, skin cells grow in a controlled and regular way. However, some newly produced cells may grow out of control and form a mass of cancer cells. Changes in the shape, size, and color of a person's mole are often the first signs of melanoma [6]. Melanoma has a black or bluish-black border; melanoma also appears as new black spots with an abnormal appearance [7]. These pigment-producing tumors are present in the surface layer of the skin (epidermis [1]). Based on the WHO reports, melanoma with 15000 cases is ranked as the fourth prevalent cancer and with 1900 cases is the ninth deadliest cancer [8].

Diagnosis of skin cancer is difficult to distinguish due to the appearance of different types of skin lesions, especially melanoma and nevi. Even with dermoscopy, a noninvasive experimental technique, the accuracy of melanoma diagnosis by dermatologists is 84-75%. Sampling, however, provides a better diagnosis that is only possible based on surgery, which can lead to an unpleasant experience for the patient.

To prevent unnecessary sampling, researchers have reviewed several noninvasive methods for diagnosing melanoma. These methods usually involve three steps: (1) skin boundary identification, (2) feature extraction, and (3) classification [9]. The border-detection process detects the tumor in skin-related images, which is essential for the accurate classification of skin lesions. The feature extraction process uses visual properties such as color, mass shape, and texture information to classify [10]. The classification process also extracts the type of skin lesions from the image features and performs classification operations.

Navid and Ghadimi [11] proposed a method for melanoma detection in the images. Edge detection and smoothing technique were used for eliminating extra scales. Then, the segmentation method was performed. During the segmentation, mathematical morphological was used for eliminating the extra information on the melanoma boundary area. The classification of the method was performed by an optimized Artificial Neural Networks (ANN) based on World Cup Optimization (WCO) algorithm to minimize the root mean square error between the network output and the desired output. The final results indicated that the suggested technique develops the method's efficacy. Recently, several research works are introduced for the early diagnosis of skin cancers [12]. For example, Sugiarti et al. [13] introduced a method for the early diagnosis of melanoma cancer. The feature extraction method of the first order was utilized for feature extraction to achieve higher precision. The classification was performed by the Artificial Neural Network (ANN). The final results indicated that that using the proposed method provides a satisfied result for the analyzed images.

The article "An Optimized Method for Skin Cancer Diagnosis Using Modified Thermal Exchange Optimization Algorithm" was published in 2021. Journal: Comput Math Methods Med.

Zhi et al. [14] presented a CAD system for early detection of skin cancer. The method uses a median filter for noise reduction. Image segmentation was done based on Convolutional Neural Network (CNN) that is optimized by Satin Bowerbird Optimization (SBO). Afterward, feature extraction and feature selection were done to extract the valuable information from the segmented image. The feature selection was based on the SBO algorithm. Final features were fed to a Support Vector Machine (SVM) classifier for final recognition. The results were validated by applying them to the American Cancer Society database and comparing them with some different techniques from the literature.

Esteva et al. [15] suggested a diagnosis technique for lesion segmentation using deep learning. The analysis of the proposed method is validated by 21 clinical images to classify them into two groups of malignant and benign classes. The study analyzed two cases: the first identified the prevalent cancers, and the other one determined the deadliest skin cancer identification. The results indicated high efficacy for the suggested method.

It is clear from the literature that several applications of the deep learning in skin cancer detection still have lots of space. Therefore, in this paper, a new optimized method has been proposed for skin lesion diagnosis with higher performance based on a new modified version of the Thermal Exchange Optimization Algorithm.

The next parts of this study are structured as follows. In “Noise Reduction from the Images,” the method of NLM based on the Yaroslavsky filter is used as a beneficial noise reduction tool. In “Image Segmentation,” the method of image segmentation which is based on the Otsu thresholding and mathematical morphology is explained. In “Methodology,” the proposed Modified Thermal Exchange Optimization Algorithm along with its application for optimal feature selection is mentioned. In “Classification,” the classification method of the study which is based on the support vector machine is stated. In “Results and Discussions,” the simulation results and their discussion are explained, and finally, the paper is concluded in “Conclusions.”

The article "An Optimized Method for Skin Cancer Diagnosis Using Modified Thermal Exchange Optimization Algorithm" was published in 2021. Journal: Comput Math Methods Med.

## 2. Noise Reduction from the Images

Preprocessing is used to correct problems in images taken that may occur during medical imaging, such as noise or light. In medical imaging, there may be disturbances due to high-frequency reception, different brightness in the field, and problems due to distant orientation, which are corrected by artificial intelligence and image processing, and usually by default on all images before the main processing. In this paper, two modifications have been used as image preprocessing to improve the system performance [16]. Due to the stochastic physical nature of imaging systems, noise in the image is unavoidable, making it difficult to perform various image processes such as segmentation, detection, and interpretation [17]. The important point during the noise reduction is that the original image and especially its details are not damaged as much as possible and the structure of the original image is preserved. Based on this, various methods have been proposed to eliminate noise. In this study, we used the newly introduced NLM method for this purpose.

The NLM filter is an extended version of the Yaroslavsky filter [18], which uses nonlocal averaging of similar pixels (pixels with a closer brightness level) to retrieve the actual amount of pixels being processed. The main advantage of the NLM method compared to this method is that it has a more stable similarity criterion in the presence of noise, because, in addition to comparing the pixels intensity levels, a neighbor of them has also a role in determining the degree of similarity. The NLM method has a good performance in reducing most noise models, especially if the noise can be distributed collectively. The NLM method is based on the weight of all the pixels in the image, in proportion to the similarity of their neighbors; in other words, the more similar the image pixel neighbors are to the pixel neighbor being processed, the higher the weight assigned to them. The amount of pixels being processed is calculated using the total weight found from the other pixels. The neighborhood criterion similarity in the NLM method is the weighted Euclidean principle with the Gaussian kernel, which is shown in Equation (1).

(1) $$\begin{array}{c} \text{d}={\left\|v\left(\eta_{i}\right)-v\left(\eta_{j}\right)\right\|}_{2\rho }^{2}=\sqrt{\overset{N}{\underset{k=1}{\sum }}w_{k}{\left(x_{ik}-x_{jk}\right)}^{2}}, \end{array}$$

where *v*(*η*_*i*_) describes the pixel neighborhood vector under process, other pixels' neighborhood vector, and ‖.‖_2*ρ*_^2^ represents the weighted Euclidean distance operator with Gaussian kernel.

The article "An Optimized Method for Skin Cancer Diagnosis Using Modified Thermal Exchange Optimization Algorithm" was published in 2021. Journal: Comput Math Methods Med.

In other words, in calculating the similarity of neighborhoods, the central pixel has a higher value, and by moving through the central pixel, the effect of the pixels decreases.

(2) $$\begin{array}{c} W\left(M_{i},M_{j}\right)=\frac{1}{Z_{i}}\exp\left(-\frac{{\left\|v\left(\eta_{i}\right)-v\left(\eta_{j}\right)\right\|}_{2\rho }^{2}}{h^{2}}\right), \end{array}$$

where

(3) $$\begin{array}{c} Z_{i}=\underset{j}{\sum }\exp\left(-\frac{{\left\|v\left(\eta_{i}\right)-v\left(\eta_{j}\right)\right\|}_{2\rho }^{2}}{h^{2}}\right) \end{array}$$

where *Z*_*i*_ is a normalization parameter that guarantees the utilized sum of weights equals 1. *h* describes the main parameter of the NLM that determines the filtering intensity. If *h* is selected small, the value of the filtering in the image is small, and the noise effect has been not removed properly, but a large value for *h* makes an overfiltering for the image, and the reconstructed image is completely blurred and devoid of fine structural details. The final equation of the NLM filter with computed weighted coefficients can be formulated as follows:

(4) $$\begin{array}{c} \text{NLM}\left(M_{i}\right)=\underset{j}{\sum }W\left(M_{i},M_{j}\right)M_{j}, \end{array}$$

Although all pixels must be weighed in retrieving each pixel image, this operation is very time-consuming, so a specific area called the search window around each pixel being processed is used for the weighting operation. As explained before, NLM is a parameter filter with the following parameters: search window radius, similarity window radius, and smoothing parameter (*h*).  Figure 1 shows a sample of noise reduction for this case.

## 3. Image Segmentation

### 3.1. Image Thresholding

The thresholding method is used to remove unnecessary information and focus on the basic information in the image. Also, if the objects in the image and the “background” have similar gray levels, this method is used to reveal hidden details in the image. Therefore, after noise reduction in the previous section, for highlighting the brain region, image thresholding has been used. One of the most popular and classic methods for finding the best threshold value is the Otsu method.

The Otsu method provides global thresholding for the input image. It uses the image histogram for maximizing the “between-class variance” of the segmented classes which consequently minimizes the “within-class variance” of the segmented classes. However, maximizing “between-class variance” needs less computational complexity than minimizing “within-class variance.” During the Otsu thresholding, we look forward to a threshold level to minimize the class variance, i.e.

(5) $$\begin{array}{c} \sigma_{\omega }^{2}\left(t\right)=\omega_{1}\left(t\right)\sigma_{1}^{2}\left(t\right)+\omega_{2}\left(t\right)\sigma_{2}^{2}\left(t\right), \end{array}$$

(6) $$\begin{array}{c} \sigma_{b}^{2}\left(t\right)=\sigma^{2}-\sigma_{\omega }^{2}\left(t\right)=\omega_{1}\left(t\right)\omega_{2}\left(t\right){\left(\mu_{1}\left(t\right)-\mu_{2}\left(t\right)\right)}^{2}, \end{array}$$

where *ω*_*i*_ signifies the probability for two separate classes with a threshold value of *t*, *σ*_*i*_^2^ describes the variance of the classes, and *μ*_*i*_(*t*) represents the mean value of the class and is updated alternately.

The article "An Optimized Method for Skin Cancer Diagnosis Using Modified Thermal Exchange Optimization Algorithm" was published in 2021. Journal: Comput Math Methods Med.

The Otsu thresholding can be briefly considered as follows:

(1) Calculate the histogram and the probabilities for each intensity level:
  (1.1) Initialize the *ω*_*i*_(0) and *μ*_*i*_(0) for all possible threshold levels
  (1.2) Update *ω*_*i*_ and *μ*_*i*_
  (1.3) Calculate *σ*_*b*_^2^(*t*)
(2) The optimal threshold is the maximum of *σ*_*b*_^2^(*t*).

### 3.2. Morphological Operations

After performing the thresholding stage, mathematical morphology has been used to abolish the spare parts of the region of interest in skin cancer images [19]. Mathematical morphology is based on applying a structural element (*e*) to the considered image. Here, a 5 × 5 identity matrix is used for structure element. In this study, mathematical filling, opening, and closing have been employed for this purpose. The first operation is to use mathematical filling. This operation is used to fill the empty holes in the threshold image. This operator can be achieved by the following equation:

(7) $$\begin{array}{c} X_{k}=\left(X_{k-1}⊕e\right)\cap A^{c},k=1,2,3\cdots , \end{array}$$

where *A* and *e* represent the area and the structure element, respectively.

After filling the holes, the mathematical opening operation has been performed to the image to eliminate the lighter details without deploying other gray surfaces. This is done by the following equation:

(8) $$\begin{array}{c} A\circ e=\left(A⊖e\right)⊕e. \end{array}$$

The last process is to perform the mathematical closing to connect the narrow parts. The formula for this operation is given below:

(9) $$\begin{array}{c} A•e=\left(A⊕e\right)⊖e. \end{array}$$

Figure 2 shows a sample for skin cancer segmentation based on the explained method.

## 4. Methodology

In this study, a new modified metaheuristic has been proposed, and then, it has been applied for providing an optimal feature selection to get better results of diagnosing.

### 4.1. The Modified Thermal Exchange Optimization Algorithm

Achieving the optimal state has been one of the most fundamental issues in the world since the creation of the universe. The scope of application of optimization-related topics is very wide. Mathematics, computer science, engineering, physics, and economics are just some of these topics. In this type of problem, the goal is to get the best decision mode from several different modes [20]. Metaheuristic algorithms can be considered one of the most important classes of optimization solutions for these types of issues. These algorithms have a lot of variety [21]. The great variety of these algorithms in solving different problems, as well as the introduction of new algorithms with different titles, has made choosing a suitable algorithm for the user who intends to use them a difficult and complex task [22]. On the other hand, each of these algorithms obtains the optimal solution with certain accuracy and speed. Therefore, it seems necessary to have a structure that can well identify the differences between these algorithms and make their comparison easier. On the other hand, the implementation of each algorithm typically requires complete knowledge of that algorithm and professional programming knowledge. Some examples of these algorithms are like the Chimp Optimization Algorithm (ChOA) [23], Black Hole (BH) [24], Crow Search Algorithm (CSA) [25], Water Strider Algorithm (WSA) [26], Ant Lion Optimizer (ALO) algorithm [27], and Thermal Exchange Optimization (MTEO) [28]. In this study, a modified version of this algorithm called the Modified Thermal Exchange Optimization (MTEO) algorithm is proposed to achieve optimal results for different parts of the diagnosis system. This TEO algorithm is a metaheuristic technique that is derived by the temperature behavior for the objects and their location which is exchanged between warm and cold parts and specifies the updated locations. More explanations are explained in the following.

The article "An Optimized Method for Skin Cancer Diagnosis Using Modified Thermal Exchange Optimization Algorithm" was published in 2021. Journal: Comput Math Methods Med.

#### 4.1.1. The Newton Law of Cooling

The Newton law of cooling states that the rate at which a body temperature changes is approximately proportional to the difference in temperature between the body and its surroundings. This was first discovered by Newton. When the temperature difference between the body and its surroundings is small, the average amount of heat exchanged between the body and its surroundings due to conduction, convection, and infrared radiation is approximately proportional to the difference in temperature of the body and the environment. Newton's law of cooling is the solution of a differential equation of the Fourier law which is formulated as follows:

(10) $$\begin{array}{c} \frac{dQ}{dt}=\alpha \times A\times \left(T_{s}-T_{a}\right), \end{array}$$

where  *Q* defines the heat, *A* signifies the body area surface which transmits heat, *α* represents the heat transfer coefficient which depends on several cases such as heat transfer mode, surface state, and object geometry, and *T*_*b*_ and *T*_*a*_ describe the body temperature and the ambient temperature.

Based on the equation, the time for losing heat is *α* × *A* × (*T*_*a*_ − *T*) *dt* which determines the change in reserved heat as the temperature falls *dT*, i.e.

(11) $$\begin{array}{c} V\times \rho \times c\times dT=-\alpha \times A\times \left(T-T_{b}\right)dt, \end{array}$$

where *c* represents the specific heat (J/kg/K), *ρ* describes the density (kg/m^3^), and *V* specifies the volume (m^3^).

Hence

(12) $$\begin{array}{c} \frac{T-T_{b}}{T_{M}-T_{b}}=\exp\left(\frac{-\alpha \times A\times t}{V\times \rho \times c}\right), \end{array}$$

where *T*_*M*_ represents the early high temperature. The above equation is correct when *α* × *A* × *t*/*V* × *ρ* × *c* is has not depended to *T*:

(13) $$\begin{array}{c} \zeta =\frac{\alpha \times A}{V\times \rho \times c}, \end{array}$$

Hence, by assuming *ζ* as a constant

(14) $$\begin{array}{c} \frac{T-T_{b}}{T_{M}-T_{b}}=\exp\left(-\zeta t\right). \end{array}$$

Accordingly

(15) $$\begin{array}{c} T=\left(T_{M}-T_{b}\right)\times \exp\left(-\gamma t\right)+T_{b}. \end{array}$$

#### 4.1.2. The Algorithm

In Thermal Exchange Optimization Algorithm, some individuals are considered cooling substances, and the other leftover individuals are considered the environment, and then, the reverse process is performed. Like any other metaheuristic algorithm, the TEO algorithm starts with initializing a definite number of randomly distributed individuals as the solution candidates. This can be presented as follows:

(16) $$\begin{array}{c} T_{i}^{0}=T_{\min}+\delta \times \left(T_{\max}-T_{\min}\right),\\ i=1,2,\cdots ,n, \end{array}$$

where *T*_*i*_^0^ describes the initial population of the algorithm for the *i*^th^ object, *δ* represents a random value limited in the range [0, 1], and *T*_min_ and *T*_max_ describe the minimum and maximum boundaries.

The cost value of all randomly generated individuals is then evaluated to indicate the cost of each algorithm. Then, the best *T* candidate vector positions have been stored as thermal memory (TM) to employ for developing the algorithm performance with less complexity. Some best TM candidates are then added to the individuals, and the same numbers of them that have the worst values are removed. Therefore, individuals have two equal types of environment, and the heat and cooling transfer objects can be seen in Figure 3.

The article "An Optimized Method for Skin Cancer Diagnosis Using Modified Thermal Exchange Optimization Algorithm" was published in 2021. Journal: Comput Math Methods Med.

To get a better conception, *T*_1_ defines the environment object for *T*_(*n*/2)+1_ cooling object, and contrariwise. If the object gives a lower value than *ζ*, the temperature exchanges gradually. In this situation, *ζ* has been achieved as follows:

(17) $$\begin{array}{c} \gamma =\frac{\text{Cos }\left(\text{object}\right)}{\text{Cos }\left(\text{worst object}\right)}. \end{array}$$

This algorithm uses time as another significant term for the simulation. This term directly depends on iteration number. This can be mathematically formulated as follows:

(18) $$\begin{array}{c} t=\frac{\text{iteration}}{\mathrm{Max}.\text{iteration}}. \end{array}$$

For increasing the global searching in the algorithm, environmental temperature changing has been considered that can be considered as follows:

(19) $$\begin{array}{c} T_{i}^{e}=\left(1-\left(m_{1}+m_{2}\times \left(1-t\right)\times \mathrm{rand}\right)\right)\times {T_{i}^{\prime }}^{e}, \end{array}$$

where *T*_*i*_′^*e*^ describes the previous temperature of the object modified by *T*_*i*_^*e*^ and *m*_1_ and *m*_2_ represent the control variables, respectively.

Considering the past models, the object new temperature can be mathematically updated by the following equation:

(20) $$\begin{array}{c} T_{i}^{+}=T_{i}^{e}+\left(T_{i}^{old}-T_{i}^{e}\right)\exp\left(-\zeta t\right). \end{array}$$

The final case which is considered in this algorithm is Pr. This term shows that a component changes in the cooling objects or not.

The Pr individuals have been compared with *R*(*i*) which has a random value in the range [0, 1]. If *R*(*i*) < Pr, one dimension of the *i*^th^ individual has been randomly selected, and the value is rewritten in the following:

(21) $$\begin{array}{c} T_{i,j}=T_{j}^{\min}+rnd\left(T_{j}^{\max}-T_{j}^{\min}\right)\exp\left(-\zeta t\right), \end{array}$$

where *T*_*i*,*j*_ describes the *j*^th^ variable of the individual number *i* and *T*_*j*_^min^ and *T*_*j*_^max^ represent the lower and the upper bounds of the variable number *j*, respectively. Finally, the algorithm will be terminated if stopping criteria have been met.

#### 4.1.3. Modified Thermal Exchange Optimization Algorithm

From the literature, the method is compared with DE, ECBO, CBO, PSO, GWO, GA, and lots of other optimization methods (20 other methods). The results showed that the original TEO has better convergence than most of the algorithms with a satisfied solution value. Then, the original paper concluded that TEO can be employed as a search engine in most of the optimization problems [28]. Also, it might be a source of inspiration for future algorithms or improved and hybridized with other methods. In this section, the details of the suggested modified Thermal Exchange Optimization Algorithm, named MWSA, have been presented. In a general form, metaheuristic algorithms should be efficient in two significant terms, exploitation and exploration, such that it can found an appropriate trade-off between them for better performance. The algorithm has the advantage of fast convergence and excellent local search capability, although it tends to fall into a local optima point rather than finding the global optimum [29–31]. In order to develop the algorithm efficiency by giving a proper balance between exploration and exploitation terms, a modification has been applied to it in this study. Opposition-based learning and chaos map are two modification mechanisms that are used here for improving algorithm efficiency.

The article "An Optimized Method for Skin Cancer Diagnosis Using Modified Thermal Exchange Optimization Algorithm" was published in 2021. Journal: Comput Math Methods Med.

The first mechanism, the opposition-based learning (OBL) mechanism, was first presented by Tizhoosh [32]. This mechanism contains a strong mathematical concept for improving the global searching of the algorithm. As aforementioned, the initializing step in TEO is completely random, and the aim is to find the best points in the solution space. Here, if the generated variables have a proper value close to the solution space, the proper solution will be achieved. But, if the algorithm starts with values too distant from the optimal solution, the time for finding the global value will be extended or even makes a premature convergence in some cases. The OBL is a mechanism to modify this issue by generating opposite values from the originally generated population. So, for every single solution, its original cost value and its opposite cost value have been compared, the best one will have remained, and the other will be removed. This can be mathematically formulated as follows:

(22) $$\begin{array}{c} {\hat{T}}_{i}^{+}=T_{\max}+T_{\min}-T_{i}^{+}, \end{array}$$

where ${\hat{T}}_{i}^{+}$ describes the opposite position of *T*_*i*_^+^ and *T*_min_ and *T*_max_ describe the variables upper and the lower bounds in the problem, respectively.

The new position provides a higher opportunity to get the best solution. The second mechanism is the chaos map. This mechanism utilizes chaotic conception to generate unpredictable variables instead of random variables. This mechanism accomplishes simple searches at a higher convergence rate than probability-based random searches [33]. By employing chaotic variables instead of random ones in metaheuristics, better exploration has been generated for the solution space because of the dynamic behavior of the sequence [34]. Several functions have been introduced as chaos functions [35]. This study employed a sinusoidal chaotic map function to modify the convergence speed of the TEO and make a balance between its exploitation and exploration terms. By considering the sinusoidal map in the TEO algorithm, environmental temperature changing is considered:

(23) $$\begin{array}{c} T_{i}^{e}=\left(1-\left(m_{1}+m_{2}\times \left(1-t\right)\times k_{i+1}\right)\right)\times {T_{i}^{\prime }}^{e}, \end{array}$$

(24) $$\begin{array}{c} k_{i+1}=\alpha \times k_{i}^{2}\sin\left(\pi .k_{i}\right), \end{array}$$

where *k*_*i*+1_ describes a chaotic random number made by current iteration and *k*_*i*_ describes the chaotic random number made by the previous iteration. *P* = 2.3 defines the control parameter, and the *k*_0_ is considered a random value in the range [0, 1].

The article "An Optimized Method for Skin Cancer Diagnosis Using Modified Thermal Exchange Optimization Algorithm" was published in 2021. Journal: Comput Math Methods Med.

#### 4.1.4. Algorithm Authentication

In this paper, in order to demonstrate the effectiveness of the suggested MTEO, eight standard benchmark functions have been selected which are listed in Table 1. To provide a comprehensive analysis on the optimization performance, the results of the proposed MTEO have been compared with some different new state-of-the-art metaheuristics, including the Biogeography-Based Optimizer (BBO) [36], Locust Swarm Optimization (LS) [37], Emperor Penguin Optimizer (EPO) [38], Spotted Hyena Optimize (SHO) [39], and original Thermal Exchange Optimization Algorithm [40]. Table 1 indicates the information about the utilized test functions.

The experiment environments are MATLAB 2019b, the Core™ i7-4720HQ with 1.60 GHz CPU, 16 GB RAM with Windows 10.  Table 2 indicates the parameters setting utilized for the comparative algorithms utilized in this study.

This study, considers two important measures including mean value and standard deviation value results from the applying optimization algorithms on the benchmark functions after 35 independent runs. To achieve a fair comparison between the proposed MTEO and the comparative algorithms, the population size for all of them and the iteration number are considered 100 and 200, respectively [41].  Table 3 illustrates the performance analysis of the comparison.

As can be observed from Table 3, the proposed MTEO algorithm provides the smallest value for the mean value of the benchmark functions. This shows that the proposed MTEO algorithm has the highest accuracy compared with the other algorithms. Also, the standard deviation value achieved by the algorithms shows the minimum value based on the MTEO algorithm that shows consequently the higher reliability of the proposed method against the other compared methods.

### 4.2. Feature Extraction and Selection

After segmentation of the region of interest from the input images, the main information (features) has been extracted from the images to reduce the complexity of the diagnosis process by considering only vital characteristics. In other words, feature extraction provides an easy way for demonstrating and analyzing the images. Recently, several algorithms have been performed for proper feature extraction of the images. During the feature extraction with different methods, all of the patterns in the features should be searched and determined. In this study, 20 different features are employed to extract the beneficial features from the segmented skin cancer for the diagnosis. In this study, three groups of features, i.e., geometric features, statistical features, and texture features, are utilized. In the following, the formulation of the utilized features is explained:

(25) $$\begin{array}{c} \text{Mean}=\frac{1}{MN}\overset{M}{\underset{i=1}{\sum }}\overset{N}{\underset{j=1}{\sum }}p\left(i,j\right), \end{array}$$

(26) $$\begin{array}{c} \text{Variance}=\frac{1}{MN}\overset{M}{\underset{i=1}{\sum }}\overset{N}{\underset{j=1}{\sum }}\left(p\left(i,j\right)-\mu \right), \end{array}$$

(27) $$\begin{array}{c} \text{Std}=\sqrt{\text{variance}}, \end{array}$$

(28) $$\begin{array}{c} \text{Contrast}=\overset{M}{\underset{i=1}{\sum }}\overset{N}{\underset{j=1}{\sum }}p^{2}\left(i,j\right), \end{array}$$

(29) $$\begin{array}{c} \text{Area}=\overset{M}{\underset{i=1}{\sum }}\overset{N}{\underset{j=1}{\sum }}p\left(i,j\right), \end{array}$$

(30) $$\begin{array}{c} \text{Rectangularity}=\frac{\text{Area}}{a\times b}, \end{array}$$

(31) $$\begin{array}{c} \text{Elongation}=\frac{2\sqrt{\text{Area}}}{a\sqrt{\pi }}, \end{array}$$

(32) $$\begin{array}{c} \text{Irregularity index}=\frac{4\pi \times \text{Area}}{\text{Perimete}{\text{r}}^{2}}, \end{array}$$

(33) $$\begin{array}{c} \text{Form Factor}=\frac{\text{Area}}{a^{2}}, \end{array}$$

(34) $$\begin{array}{c} \text{Eccentricity}=2a^{-1}{\left(a^{2}-b^{2}\right)}^{0.5}, \end{array}$$

(35) $$\begin{array}{c} \text{Entropy}=\overset{M}{\underset{i=1}{\sum }}\overset{N}{\underset{j=1}{\sum }}p\left(i,j\right)\log p\left(i,j\right), \end{array}$$

(36) $$\begin{array}{c} \text{Perimeter}=\overset{M}{\underset{i=1}{\sum }}\overset{N}{\underset{j=1}{\sum }}b_{p}\left(i,j\right), \end{array}$$

(37) $$\begin{array}{c} \text{Homogeneity}=\overset{M}{\underset{i=1}{\sum }}\overset{N}{\underset{j=1}{\sum }}\frac{p\left(i,j\right)}{1+\;|\;i-j\;|\;}, \end{array}$$

(38) $$\begin{array}{c} \text{Energy}=\overset{M}{\underset{i=1}{\sum }}\overset{N}{\underset{j=1}{\sum }}p^{2}\left(i,j\right), \end{array}$$

(39) $$\begin{array}{c} \text{Correlation}=\overset{M}{\underset{i=1}{\sum }}\overset{N}{\underset{j=1}{\sum }}\frac{\text{p}\left(i,j\right)-\mu_{r}\mu_{c}}{\sigma_{r}\sigma_{c}}, \end{array}$$

(40) $$\begin{array}{c} \varphi_{1}=\eta_{20}+\eta_{02}, \end{array}$$

where *b*_*p*_ signifies the external side length of the boundary pixel, *p*(*i*, *j*) represents the pixel intensity value at point (*i*, *j*), MN describes best the image size, *a* and *b* represent the major and the minor axis, respectively, and *μ* and *σ* represent the mean value and the standard deviation value, respectively.

The article "An Optimized Method for Skin Cancer Diagnosis Using Modified Thermal Exchange Optimization Algorithm" was published in 2021. Journal: Comput Math Methods Med.

Because of the higher volume of feature information and the presence of some useless features, some of these features should be then eliminated before the classification stage. This is done by using a method, called feature selection. To achieve an optimal diagnosis system, the suggested modified Thermal Exchange Optimization Algorithm has been utilized that is explained in the following.

Feature selection is the process of reducing the data dimension by choosing the best features and eliminating the others. Furthermore, however, some features are useless, but once they blend with other features, they have been beneficial. This study uses a definite cost function where by minimizing it, the optimal features can be selected. The cost function is formulated in the following:

(41) $$\begin{array}{c} CF=\frac{\left(TP\times TN\right)-\left(FP\times FN\right)}{\sqrt{\left(TN+FP\right)\times \left(TP+FP\right)\times \left(TP+FN\right)\times \left.\left(TN+FN\right)\right)}}, \end{array}$$

where *TP*, *FP*, *TN*, and *FN* represent the true positive, false positive, true negative, and false negative, respectively.

The main idea is to minimize the above function. This is performed by the proposed modified Thermal Exchange Optimization Algorithm.

## 5. Classification

The classification in this study is based on the Support Vector Machine (SVM). The SVM consists of a set of points in the *n*-dimensional space of data which indicates the class boundaries and organizes them and can be altered with the rearrangement of one of these two cases. The SVM provides the best results for separating the data with the criterion for placement of the support vectors. This classifier organizes the best separation surface by the following equation:

(42) $$\begin{array}{c} y=\mathrm{sgn}\left(\overset{N}{\underset{i=1}{\sum }}y_{i}\alpha_{i}K\left(x,x_{i}\right)+b\right), \end{array}$$

where *K*(*x*, *x*_*i*_) describes a kernel function, *x* signifies a test set vector with *d* dimensions, *x*_*i*_ describes the *i*^th^ training set vector, *y* represents the output class by labeling -1 or 1, *N* is the number of the training set, and *b* and *α* = [*α*_1_ ⋯ *α*_*N*_] represent the model parameters, respectively.

The article "An Optimized Method for Skin Cancer Diagnosis Using Modified Thermal Exchange Optimization Algorithm" was published in 2021. Journal: Comput Math Methods Med.

The present study uses SVM for the classification of the extracted features achieved by the feature selection in the previous stage into two parts of healthy and cancerous groups.

## 6. Results and Discussions

The main purpose of this study is to present a computer-aided automatic method for optimal diagnosis of skin cancer from the dermoscopy images. The idea is to utilize a metaheuristic-based method to achieve the best feature selection, and consequently the best diagnosis.

### 6.1. Database

To validate the proposed skin cancer diagnosis system, the so-called American Cancer Society (ACS) database has been employed. This database contains 68 pairs of XLM and TLM images that are collected from the Nevoscope system. 51 XLM images and 60 TLM images have been manually classified by a dermatologist since other images do not show pigmentation [42]. Therefore, the validation has been based on comparing our results with these manually segmented results. For giving less complexity to the analysis, all of the images are resized to 256 to 256 pixels. Some examples of this database are given in Figure 4 [43].

### 6.2. Simulation Results

The present study in this subsection has been verified on the ACS database, and the results have been validated based on some different state-of-the-art techniques. Simulations have been validated by the MATLAB 2019b environment with the following hardware configuration: Core™ i7-4720HQ 1.60 GHz with 16 GB RAM. The overall procedure of the suggested method is illustrated in Figure 5.

The present study uses 85% of the data for training and 15% for testing the data. The training stage is based on applying 750 iterations and is iterated 20 times independently to achieve a guaranteed result. Five measurement indicators including PPV, NPV, specificity, accuracy, and sensitivity are used for validation that is formulated as follows:

(43) $$\begin{array}{c} \text{PPV}=\frac{\text{correctly detected skin cancer cases}}{\text{detected skin cancer cases }}, \end{array}$$

(44) $$\begin{array}{c} \text{NPV}=\frac{\text{correctly detected healthy skin cases}}{\text{detected healthy skin cases}}, \end{array}$$

(45) $$\begin{array}{c} \text{Specificity}=\frac{\text{correctly detected healthy skin cases}}{\text{total healthy skin cases }}, \end{array}$$

(46) $$\begin{array}{c} \text{Accuracy}=\frac{\text{correctly detected cases}}{\text{total cases}}, \end{array}$$

(47) $$\begin{array}{c} \text{Sensitivity}=\frac{\text{correctly detected skin cancer cases}}{\text{Total skin cancer cases }}. \end{array}$$

To give a fair analysis on the proposed method, its results have been compared with some different state-of-the-art methods including the Particle Swarm Optimization- (PSO-) based method [44], m-Skin Doctor [45], GFAC [46], ANN [47], and Genetic Algorithm (GA) [42]. The results of the validation are tabulated in Table 4.

The article "An Optimized Method for Skin Cancer Diagnosis Using Modified Thermal Exchange Optimization Algorithm" was published in 2021. Journal: Comput Math Methods Med.

It can be observed from Table 4 that the proposed optimized methodology with 92.79% accuracy has the highest precision against the other comparative methods. Similarly, with 90.99% sensitivity, it has proper reliability compared with the other methods. This is also proved for the specificity, NPV, and PPV compared with the others. The higher value of NPV and PPV including 93.69% and 85.58%, respectively, which are the highest among the comparative methods, provides the higher prevalence of the condition to diagnose the likelihood of a test cancer diagnosis system. Finally, the better results of the sensitivity and specificity for the proposed method indicate the suggested method's higher prevalence-independent results.

## 7. Conclusions

Skin cancer is one of the most dangerous diseases among different cancers in the world. However, early detection of this disease can be so beneficial for cancer treatment. In the present study, a new hierarchical methodology was proposed for the optimal diagnosis of skin cancer from dermoscopy images. According to the suggested method, after performing noise reduction of the input dermoscopy images, the considered area has been segmented based on a simple Otsu. Then, feature extraction has been performed to the processed image to extract valuable features from the images. To provide an optimized result, the best features have been selected by a modified metaheuristic method, called the Modified Thermal Exchange Optimization Algorithm to modify the network performance in terms of precision and consistency. Final results were obtained by applying support vector machine as the final classifier. To give a proper validation, the results of the proposed method were applied to the American Cancer Society (ACS) database, and its results were compared with some different methods including Particle Swarm Optimization- (PSO-) based method, m-Skin Doctor, GFAC, ANN, and Genetic Algorithm (GA). The final results indicated that according to different measurement indicators, the proposed methodology has the best results for the other compared methods. As can be observed from the explanations, the proposed method has good results for skin cancer detection. However, this can be an inspiration to our future work to use different hybrid and developed versions of different new computational intelligence algorithms like the Monarch Butterfly Optimization (MBO) [48], Earthworm Optimization Algorithm (EWA) [49], Elephant Herding Optimization (EHO) [50], Moth Search (MS) algorithm [51], Slime Mold Algorithm (SMA) [52], and Harris hawks optimization (HHO) [53] to improve the system efficiency.

The article "An Optimized Method for Skin Cancer Diagnosis Using Modified Thermal Exchange Optimization Algorithm" was published in 2021. Journal: Comput Math Methods Med.

## Figures and Tables

**Figure 1:** Image noise reduction: (a) before and (b) after processing.

**Figure 2:** A sample for skin cancer segmentation based on the explained method: (a) input image and (b) segmented.

**Figure 3:** The pairs of environment and the heat and cooling transfer objects.

**Figure 4:** Some examples of the American Cancer Society (ACS) database [43].

**Figure 5:** The pipeline of the proposed methodology.

**Table 1:** The information about the utilized test functions.

No.	Test function	Minimum value	Boundary
1	$F_{1}=\overset{N}{\underset{n=1}{\sum }}x_{n}^{2}$	0	−∞≤*x* ≤ ∞
2	$F_{2}=\overset{N-1}{\underset{n=1}{\sum }}\left(100\times {\left[x_{n+1}-x_{n}^{2}\right]}^{2}+{\left[1-x_{n}\right]}^{2}\right)$	0	−∞≤*x*_*n*_ ≤ ∞
3	$F_{3}=\overset{N}{\underset{n=1}{\sum }}\left|x_{n}\right|-10\cos\left(\sqrt{\left|10x_{n}\right|}\right)$	0	−∞≤*x*_*n*_ ≤ ∞
4	*F*_4_ = *x*sin(4*x*) + 1.1*y*sin (2*y*)	-18.5547	0 ≤ *x*, *y* ≤ 10
5	$F_{5}=\left[\overset{N}{\underset{n=1}{\sum }}{nx}_{n}^{4}\right]+N_{n}\left(0,1\right)$	Varies	−∞≤*x* ≤ ∞
6	$F_{6}=10N+\overset{N}{\underset{n=1}{\sum }}\left[x_{n}^{2}-10\cos\left(2\pi x_{n}\right)\right]$	0	−∞≤*x*_*n*_ ≤ ∞
7	$F_{7}=1+\overset{N}{\underset{n=1}{\sum }}\frac{x_{n}^{2}}{4000}-\overset{N}{\underset{n=1}{\prod }}\cos\left(x_{n}\right)$	0	−∞≤*x*_*n*_ ≤ ∞
8	$F_{8}=\frac{1}{2}+\frac{\sin^{2}\sqrt{x^{2}+y^{2}}-0.5}{1+0.1\left(x^{2}+y^{2}\right)}$	-0.5231	−∞≤*x*, *y* ≤ ∞

**Table 2:** The parameters setting utilized for the comparative algorithms utilized in this study.

Algorithm	Parameter	Value	Algorithm	Parameter	Value
BBO [36]	*P*_habit_	1	EPO [38]	$\overset{⟶}{A}$	[-1.5, 1.5]
	*P*_imig_	[0,1]		*T*′	[1, 1000]
	Step size	1		*M*	2
	*E*	1		*f*	[2, 3]
	*I*	1		S	[0, 1.5]
	*P*_mutation_	0.005		*l*	[1.5, 2]
LS [37]	*F*	0.6	SHO [39]	$\overset{⟶}{M}$	[0.5, 1]
	*L*	1		$\overset{⟶}{h}$	[5, 0]
	*g*	20			

**Table 3:** The performance analysis of the comparative algorithms applied to studied standard benchmarks.

Algorithm		BBO [36]	LS [37]	EPO [38]	SHO [39]	TEO	MTEO
Function							
*f*_1_	Min	2.615*e*-25	1.1100*e*-29	-3.2688*e*-26	2.3086*e*-27	2.4400*e*-30	9.2082*e*-32
	Std	1.448*e*-20	3.3826*e*-28	4.0754*e*-27	1.8827*e*-28	1.0062*e*-32	3.2681*e*-33

*f*_2_	Min	6.0652*e*-4	8.3420*e*-3	5.6024*e*-3	1.4527*e*-4	2.4352*e*-5	7.6700*e*-5
	Std	4.1073*e*-5	3.0718*e*-4	1.0056*e*-4	2.4807*e*-5	3.0537*e*-6	1.0142*e*-5

*f*_3_	Min	-6.1442	-9.0464	-9.86	-8.0826	-9.86	-9.86
	Std	0.31	0.42	0.23	0.11	0.11	0.06

*f*_4_	Min	-6.1735	-17.020	-16.0035	-15.2816	-17.0095	-17.0572
	Std	3.015	1.183	2.280	4.089	1.520	0.980

*f*_5_	Min	12.35*e*-10	1.486*e*-15	3.0765*e*-8	4.0802*e*-8	1.7085*e*-22	2.6827*e*-23
	Std	7.831*e*-11	3.0862*e*-16	1.1832*e*-9	5.4403*e*-9	3.7786*e*-24	6.0826*e*-25

*f*_6_	Min	5.165*e*-10	3.1842*e*-11	1.0856*e*-20	1.0846*e*-9	3.0008*e*-20	4.5013*e*-22
	Std	8.186*e*-11	2.4253*e*-13	5.1738*e*-22	4.7080*e*-11	1.2058*e*-21	2.5387*e*-23

*f*_7_	Min	3.512*e*-14	2.2621*e*-9	4.0305*e*-8	2.6517*e*-10	1.5670*e*-9	7.2837*e*-16
	Std	1.056*e*-15	3.0856*e*-11	3.8253*e*-9	2.1825*e*-12	2.0834*e*-10	3.1175*e*-18

*f*_8_	Min	0.0056	-0.1361	-0.2381	-0.4735	-0.4680	-0.4162
	Std	0.542	0.356	0.274	0.704	0.141	0.089

The article "An Optimized Method for Skin Cancer Diagnosis Using Modified Thermal Exchange Optimization Algorithm" was published in 2021. Journal: Comput Math Methods Med.

**Table 4:** The validation results of the compared method for skin cancer diagnosis.

Method	Performance metric				
	NPV	PPV	Specificity	Accuracy	Sensitivity
PSO	93.69	89.19	88.29	88.29	90.99
m-Skin Doctor	83.87	65.76	61.26	81.98	83.78
GFAC	88.28	77.48	82.88	86.48	89.19
ANN	82.88	58.56	56.76	67.57	81.98
GA	85.58	74.77	79.28	81.08	79.28
Proposed method	93.69	85.58	89.19	92.79	90.99

## Data Availability

The authors of this paper thank the contributors of the PH2 skin cancer database. The major part of the data considered to support the findings of this study is collected from the PH2 database.
